The article "Alpha-Ketoglutarate Alleviates Neuronal Apoptosis Induced by Central Insulin Resistance through Inhibiting S6K1 Phosphorylation after Subarachnoid Hemorrhage" was published in 2022. Journal: Oxid Med Cell Longev.

# Alpha-Ketoglutarate Alleviates Neuronal Apoptosis Induced by Central Insulin Resistance through Inhibiting S6K1 Phosphorylation after Subarachnoid Hemorrhage

**DOI:** 10.1155/2022/9148257

**Published:** 2022-08-25

**Authors:** Peng-Fei Ding, Qi Zhu, Bin Sheng, Heng Yang, Hua-Jie Xu, Tao Tao, Zheng Peng, Xiang-Xin Chen, Xiao-Jian Li, Yan Zhou, Hua-Sheng Zhang, Yong-Yue Gao, Zong Zhuang, Chun-Hua Hang, Wei Li

**Affiliations:** ^1^Department of Neurosurgery, Nanjing Drum Tower Hospital Clinical College of Nanjing Medical University, Nanjing, 210008 Jiangsu, China; ^2^Department of Neurosurgery, Nanjing Drum Tower Hospital, The Affiliated Hospital of Nanjing University Medical School, 321 Zhongshan Road, Nanjing 210008, China

## Abstract

Neuronal apoptosis after subarachnoid hemorrhage (SAH) is believed to play an important role in early brain injury after SAH. The energy metabolism of neuron is closely related to its survival. The transient hyperglycemia caused by insulin resistance (IR) after SAH seriously affects the prognosis of patients. However, the specific mechanisms of IR after SAH are still not clear. Studies have shown that *α*-KG takes part in the regulation of IR and cell apoptosis. In this study, we aim to investigate whether *α*-KG can reduce IR after SAH, improve the disorder of neuronal glucose metabolism, alleviate neuronal apoptosis, and ultimately play a neuroprotective role in SAH-induced EBI. We first measured *α*-KG levels in the cerebrospinal fluid (CSF) of patients with SAH. Then, we established a SAH model through hemoglobin (Hb) stimulation with HT22 cells for further mechanism research. Furthermore, an in vivo SAH model in mice was established by endovascular perforation. Our results showed that *α*-KG levels in CSF significantly increased in SAH patients and could be used as a potential prognostic biomarker. In in vitro model of SAH, we found that *α*-KG not only inhibited IR-induced reduction of glucose uptake in neurons after SAH but also alleviated SAH-induced neuronal apoptosis. Mechanistically, we found that *α*-KG inhibits neuronal IR by inhibiting S6K1 activation after SAH. Moreover, neuronal apoptosis significantly increased when glucose uptake was reduced. Furthermore, our results demonstrated that *α*-KG could also alleviate neuronal apoptosis in vivo SAH model. In conclusion, our study suggests that *α*-KG alleviates apoptosis by inhibiting IR induced by S6K1 activation after SAH.

## 1. Introduction

Subarachnoid hemorrhage (SAH) is a common neurosurgical emergency, in which 85% of cases are caused by aneurysms [1]. Kusaka et al. proposed early brain injury (EBI), including cellular apoptosis, neuroinflammation, and brain edema [2], among which neuronal apoptosis was thought to play an important role in EBI [3]. Previous studies have proved that inhibition of neuronal apoptosis after SAH can improve neural function and reduce EBI [4, 5]. Therefore, targeted inhibition of neuronal apoptosis may be a reliable treatment for EBI.

The article "Alpha-Ketoglutarate Alleviates Neuronal Apoptosis Induced by Central Insulin Resistance through Inhibiting S6K1 Phosphorylation after Subarachnoid Hemorrhage" was published in 2022. Journal: Oxid Med Cell Longev.

The survival of cells is closely related to energy metabolism. Glucose transport and metabolism can serve as important regulatory points in the early apoptotic cascade [6]. A number of studies have shown that SAH patients with or without a history of diabetes will have transient hyperglycemia after bleeding, which seriously affects the prognosis [7–9]. Researchers proposed that insulin resistance (IR) after SAH was the direct cause of this phenomenon [9, 10], but the mechanisms remain unclear. Neurons are the ultimate beneficiaries of glucose transport [11–13], consuming 80%-85% of ATP required by brain [14] and widely expressing glucose transporter isoforms GLUT3 and GLUT4 [15]. Membrane translocation of GLUT4 in muscle and adipose tissue is insulin-dependent. IR in neurodegenerative disorders of ageing (NDAs) has also shown decreased glucose uptake in neurons [16, 17]; hence, Cunnane et al. speculate that GLUT 4 in neurons may also be insulin-dependent [13].

Studies have found that insulin selectively acts through IRS1 in adult cerebellar cortex and hippocampus [18]. Normally, binding of insulin receptors to insulin results in tyrosine phosphorylation of the receptor itself, which promotes IRS1 tyrosine phosphorylation at multiple sites, and then acts through the PI3K/AKT/mTOR pathway [19]. S6K1 is a serine/threonine protein kinase downstream of mTOR in the insulin signaling pathway, which plays an important role in driving IR [20]. S6K1 deficiency has been verified to prevent age- and diet-related obesity while enhancing insulin sensitivity. In addition, the activity of S6K1 and p-IRS1 (Ser636/S639) levels significantly increased in wild-type mice receiving a high-fat diet as well as in two obesity genetic models [21]. Abnormal serine phosphorylation occurs in neuron IRS1 during IR, so p-IRS1 (Ser636/639)/IRS1 can be used as a marker of peripheral and cerebral IR [22–24].

ATP required by neurons is mainly produced by oxidative phosphorylation of glucose through the tricarboxylic acid (TCA) cycle in mitochondria [13]. As an important intermediate metabolite of TCA, alpha-ketoglutaric acid (*α*-KG) regulates TCA [25] and participates in a variety of cellular metabolic pathways [26]. Recent studies have shown that oral *α*-KG could improve IR induced by obesity and decrease blood glucose in mice [27, 28]. Moreover, *α*-KG can promote glucose uptake and increase cell viability by upregulating GLUT1 under low glucose conditions [29]. Thus, inhibition of IR promotes membrane translocation of the GLUT protein family and furthermore increases cellular glucose uptake, which may account for the reasons why *α*-KG inhibits apoptosis [30].

The article "Alpha-Ketoglutarate Alleviates Neuronal Apoptosis Induced by Central Insulin Resistance through Inhibiting S6K1 Phosphorylation after Subarachnoid Hemorrhage" was published in 2022. Journal: Oxid Med Cell Longev.

In conclusion, we hypothesized that IR after SAH could further lead to neuronal apoptosis by affecting neuronal glucose metabolism, and *α*-KG could rescue this process by reducing IR in brain tissue. Consequently, we examined *α*-KG levels in cerebrospinal fluid of SAH patients and verified the possible mechanisms in vitro. Besides, the protective effects of *α*-KG after SAH were also researched both in vitro and in vivo.

## 2. Methods and Materials

### 2.1. CSF Collection and Experimental Analysis

We collected CSF samples from SAH patients admitted to the Department of Neurosurgery at Nanjing Drum Tower Hospital, the Affiliated Hospital of Nanjing University Medical School, from July 2019 to April 2021. All samples are the leftover of CSF samples acquired for normal diagnostic purpose. The following inclusion criteria were used: (1) age between 18 and 80 years; (2) diagnosis of spontaneous SAH; and (3) unbearable headache, increased intracranial pressure, or fever of unknown cause indicating the need for a lumbar puncture. Exclusion criteria were as follows: (1) age less than 18 or more than 80 years old; (2) the duration from ictus to admission is more than 24 h; and (3) with no need for lumbar puncture or refusal of the procedure. Consent forms were signed by the patients or direct relatives involved in this study. Fifty CSF samples at 1–3 days (C1) after SAH and 21 samples at 5–7 days (C2) after SAH were collected by lumbar puncture. There are 21 patients with both C1 and C2. Biological samples were centrifuged (2500 rpm for 30 min), and supernatants were aliquoted and frozen at –80°C for further analysis. *α*-KG levels were quantified using an enzyme-linked immunosorbent assay kit (AiFang biological, China). Written informed consent was received from participants or valid proxies prior to inclusion in the study. The study was approved by the Research Ethics Committee of Nanjing Drum Tower hospital (No. 2020-041-01).

### 2.2. Clinical Data

Demographics and past medical history (hypertension) were recorded. SAH severity was measured according to the Hunt-Hess grading scale. The digital subtraction angiography and the location of aneurysm information were also collected. The blood glucose level was collected on the same day or the nearest day to lumbar puncture. And the last blood glucose before hospital discharge (at least 7 days post SAH) was defined as the blood glucose baseline since we know the glucose burden of SAH patients returns to normal at around 7 days post SAH [7, 10]. All blood glucose levels were obtained as routine hospital examinations. Outcomes were assessed by Modified Rankin Scale (MRS) at 3 months after hospital discharge by the patients or close relatives. Good outcome was defined as MRS 0 to 2, and poor outcome was defined as MRS 3 to 6.

The article "Alpha-Ketoglutarate Alleviates Neuronal Apoptosis Induced by Central Insulin Resistance through Inhibiting S6K1 Phosphorylation after Subarachnoid Hemorrhage" was published in 2022. Journal: Oxid Med Cell Longev.

### 2.3. In Vitro Model of SAH

Insulin receptors are highly expressed in the brain, mainly distributed in the cortex, hippocampus, and hypothalamus [31]. Therefore, we chose the mouse hippocampal neuron HT22 cells. The cell lines were purchased from Shanghai Institute of Cell Biology, Chinese Academy of Sciences. The culture condition was DMEM medium containing 10% fetal bovine serum. Cells were incubated in incubators at 37°C and 5% CO_2_. Bovine hemoglobin (Sigma, USA) was dissolved in complete medium (25 *μ*mol/L) and incubated to establish SAH model in vitro.

### 2.4. Cell Viability Assay by Cell Counting Kit-8

HT22 cells were cultured in 96-well plates at a density of 1 × 10^4^ cells per well. After proper treatments, the medium was replaced completely with normal culture medium and 10 *μ*L CCK8 (Dojindo Laboratories, Japan). After a 1 h incubation at 37°C, the absorbance was detected at 450 nm in a microplate reader (Thermo, United states). The relative cell viability was calculated according to the manual. Conditioned medium (CM) was collected from treated HT22 cells and filtered through a 0.22 *μ*m filter.

### 2.5. Preparation of Palmitic Acid

Palmitic acid (PA) is a classical inducer of insulin resistance and has no cytotoxicity at concentrations below 200 *μ*M [32]. The analytical balance was used to weigh 0.0278 g PA powder and dissolve it in 1 mL double distilled water. Repeatedly shock to dissolve in 55-60°C water bath, 0.1 m palmitic acid mother liquor; 1.9 g bovine blood albumin (BSA) powder was accurately weighed and dissolved in 19 mL double distilled water to obtain 10% BSA solution. Transfer 0.1 M palmitic acid mother solution to 10% BSA solution to obtain 5 mM palmitic acid solution. DMEM medium containing 10% FBS was diluted to 200 *μ*M before use.

### 2.6. Cell Membrane Protein Extraction

Cells were cultured in 6-well plates and washed with PBS after absorbing the medium. The cells were treated with a cellular digest containing EDTA but without trypsin so that they did not stick to the wall and then dispersed the medium by pipetting over the cell layer surface several times. Cells were collected by centrifugation, supernatant was removed, and cell precipitation was left for later use. Steps followed manufacturer's instructions (Beyotime, P0033).

The article "Alpha-Ketoglutarate Alleviates Neuronal Apoptosis Induced by Central Insulin Resistance through Inhibiting S6K1 Phosphorylation after Subarachnoid Hemorrhage" was published in 2022. Journal: Oxid Med Cell Longev.

### 2.7. Real-Time PCR

Total RNA was prepared with TRIzol (Invitrogen, USA) according to the manufacturer's instructions. cDNA was reverse transcribed from mRNA with reverse transcription mix (Vazyme, Nanjing). qPCR was performed with SYBR Green mix (Roche, Switzerland) using the PCR system (Applied Biosystems, USA). The results were analyzed with the 2 − *ΔΔ*Ct method. Primers used in qPCR are listed in Table 1.

### 2.8. Western Blot

Cultured cells were lysed with RIPA (Thermo Scientific, USA) and protease inhibitor (Roche, Switzerland) and 1% phosphatase inhibitor (Sigma, USA) on ice. Protein quantification was performed with a bicinchoninic acid protein assay kit (Beyotime, China). The same mass of protein was loaded onto SDS-PAGE gels and then transferred to polyvinylidene difluoride membranes (Millipore, USA). Membranes were blocked with 1% BSA for 1 h at room temperature and incubated with primary antibody overnight at 4°C and then conjugated secondary antibody 1 h at room temperature. Incubate the blot with the working solution for 1 min when using standard ECL substrates or 5 min. Bands were analyzed using ImageJ. Antibodies used in WB are listed in Table 1.

### 2.9. Measurement of Glucose Uptake

2-NBDG is a fluorescently labeled 2-deoxyglucose analogue that competitively inhibits with D-glucose and can therefore be used as a tracer for glucose metabolism in cells (Amgicam, AJCI4820). The cells were cultured in 12-well plates, washed with PBS for 3 times, and incubated with 100 *μ*M at 37°C for 20 min, then washed with PBS for 3 times. Three regions were randomly selected from each well for observation under fluorescence microscope, and the experiment was repeated three times. The average fluorescence intensity was calculated by ImageJ, and each hole was repeated 3 times with 3 holes in each group.

### 2.10. Flow Cytometry

The cells were cultured in 12-well plates, digested with trypsin without EDTA, and collected after digestion. Centrifugation was performed at 1000 rpm at 4°C for 5 min, and the supernatant was discarded. The cells were washed twice with precold PBS at 1000 rpm and centrifuged at 4°C for 5 min, and the supernatant was discarded. The cells were suspended by 100 *μ*M 1x binding buffer. Annexin V-FITC 5 *μ*M and PI staining solution 5 *μ*M were added and incubated at room temperature for 10 min (Vazyme, a211-01), protected from light. Add 400 *μ*M 1x binding buffer and mix. C6 flow cytometry was used for detection, and FlowJo (version 10) was used for analysis.

### 2.11. Caspase-3 Activity Assay

Caspase-3 activity was measured by using a caspase-3 activity kit (Beyotime, C1115). After cell lysates were incubated with Ac-LEVD-pNA for 2 h at 37°C, the samples were read at 405 nm. Caspase-3 activity is expressed as the fold of enzyme activity compared to cells without Hb stimulation.

The article "Alpha-Ketoglutarate Alleviates Neuronal Apoptosis Induced by Central Insulin Resistance through Inhibiting S6K1 Phosphorylation after Subarachnoid Hemorrhage" was published in 2022. Journal: Oxid Med Cell Longev.

### 2.12. In Vitro S6K1 Assay

S6K1 activity was measured by using an ADP-Glo™ kinase kit (Promega, V9611). Briefly, recombinant human S6K1 (25 ng per well) was mixed with dimethyl *α*-KG (DMKG; Sigma, 349631) or PF-4708671 (10 *μ*M) 20 minutes on ice. S6K1 substrate and ATP mix (25 *μ*M, final concentration) were added and incubated at room temperature for 60 min. ADP-Glo reagent (25 *μ*L per well) was then added and incubated for 40 min. After the addition of the kinase detection buffer (50 *μ*L per well) and incubation for 30 min, record luminescence.

### 2.13. Mice and Model

A total of 31 adult male C57BL/6 mice (6–8 weeks old, 20–25 g) were purchased from Animal Core Facility of Nanjing Medical University. Animal care and experiments were performed in accordance with the Guide for the Care and Use of Laboratory Animals of the National Institutes of Health. All studies were reviewed and approved by the Animal Experiment Administration Committee of the Nanjing Drum Tower Hospital (No. 2022AE01007).

The endovascular perforation method was used to establish SAH models in this study. Animals were anesthetized with 2% isoflurane inhalation for induction and maintenance. After satisfactory anesthesia, the external carotid artery (ECA), internal carotid artery (ICA), and common carotid artery were fully exposed, and after distal ligation of ECA, a blunt 6-0 nylon suture was inserted in the ECA and advanced through the ICA for about 1.0 cm. For the sham group, all procedures were the same except for the puncture of the ECA. All mice were given 0.5 mL of normal saline intraperitoneally after surgery. We used a modified Garcia score to exclude animals which scored ≤6 or ≥15 on postoperative day.

As reported in previous article [27, 28], oral *α*-KG administration can improve IR. We chose 3 consecutive days of intragastric administration at a dose of 1% DMKG in 0.5 mL normal saline twice a day after SAH model made.

Animals were randomly divided into three groups: sham group (*n* = 6), SAH group (*n* = 6), and SAH+DMKG group (*n* = 6). Three mice of each group were used to extract perifocal tissue protein for Western blot, and three mice of each group were used to obtain whole brain for frozen sections.

### 2.14. TUNEL Assays

TUNEL assays were performed with the one-step TUNEL kit according to the manufacturer's instructions (Beyotime, C1090). We first incubated with the primary antibody anti-NeuN (Cell Signaling Technology, 94403S) overnight and incubated with the corresponding secondary antibody for 1 h. Then, we added the TUNEL mixture followed the instruction. The whole-brain NeuN^+^ TUNEL^+^/NeuN^+^ proportion was analyzed with ImageJ (*n* = 3 brains). NeuN^+^ TUNEL^+^/NeuN^+^ proportion = (area (NeuN^+^ cells) + area (TUNEL^+^ cells) − area (positive cells in merge figure))/area (NeuN^+^ cells) × 100% [33].

The article "Alpha-Ketoglutarate Alleviates Neuronal Apoptosis Induced by Central Insulin Resistance through Inhibiting S6K1 Phosphorylation after Subarachnoid Hemorrhage" was published in 2022. Journal: Oxid Med Cell Longev.

### 2.15. Statistical Analysis

All data were expressed as the mean ± standard error of the mean (SEM). All data were first tested for normality and the homogeneity of variance. Statistical analysis was performed using Prism 8.02 (GraphPad Software, USA), SPSS 22.0 (SPSS Inc., Chicago, IL, USA), and MedCalc 20 (MedCalc Software, Mariakerke, Belgium). Categoric variables were expressed as frequencies and percentages, and comparisons between groups were performed using the *χ*^2^ or Fisher tests. Two-tailed Student's *t*-test was used to assess differences between two groups, and one-way ANOVA followed by Tukey's test was used for comparisons of more than two groups if met the homogeneity of variance. If not met the homogeneity of variance, Kruskal-Wallis 1-way ANOVA was used for comparisons of more than two groups. The Spearman rank correlation test was used to test the correlation of *α*-KG and MRS and Hunt-Hess score. Receiver operating characteristic (ROC) curve analysis was carried out to determine the area under the curve (AUC). The AUC differences between *α*-KG and glucose were performed by a *z*-test. *P* < 0.05 was considered statistically significant.

## 3. Results

### 3.1. After SAH, *α*-KG Increased Continuously in CSF

Patients' characteristics are listed in Table 2. Compared with the control group, *α*-KG levels in cerebrospinal fluid in SAH patients continued to increase 0-7 days after hemorrhage (Figure 1(a)) (control vs. C1, 5.09 ng/mL (3.23-6.95) vs. 15.81 ng/mL (10.02-21.59); control vs. C2, 5.09 ng/mL (3.23-6.95) vs. 24.01 ng/mL (18.71-29.32); C1 vs. C2, 15.81 ng/mL (10.02-21.59) vs. 24.01 ng/mL (18.71-29.32)). Besides, the 21 patients who both have C1 and C2 were taken paired test (C1 vs. C2, 15.00 ng/mL (11.08–18.91) vs. 24.01 ng/mL (18.71-29.32)). The blood glucose level increased significantly at 1 to 3 days and fell back at 5 to 7 days, presenting a transient increase (Figure 1(b)) (baseline vs. B1, 5.32 mmol/L (3.97-6.68) vs. 6.70 mmol/L (5.10-8.30); B1 vs. B2, 6.70 mmol/L (5.10-8.30) vs. 5.49 mmol/L (4.64-6.34); baseline vs. B2, 5.32 mmol/L (3.97-6.68) vs. 5.49 mmol/L (4.64-6.34)). Besides, the 21 patients who both have B1 and B2 were taken paired test (B1 vs. B2, 7.07 mmol/L (5.55-8.59) vs. 5.49 mmol/L (4.64-6.34)).

### 3.2. *α*-KG Predicted the Prognosis of SAH Patients

*α*-KG levels in C1 could predict patient outcomes (Figure 1(c)) (good outcome vs. poor outcome, 14.53 ng/mL (9.03–20.03) vs. 20.32 ng/mL (15.84-24.81)). It was also shown that *α*-KG levels in C1 positively correlated with MRS score (*r* = 0.395, *P* < 0.01), rather than Hunt-Hess score (*r* = −0.11, *P* = 0.943) (Figure 1(g)). Meanwhile, glucose level in B1 can also predict the prognosis of patients (Figure 1(e)) (good outcome vs. poor outcome, 6.42 mmol/L (5.01–7.84) vs. 7.68 mmol/L (5.79-9.57)), whereas *α*-KG levels in C2 did not differ between the two groups (Figure 1(d)) (good outcome vs. poor outcome, 23.80 ng/mL (18.12-29.48) vs. 24.92 ng/mL (21.16–28.68)). Glucose levels in B2 were not different between the two groups (Figure 1(f)) (good outcome vs. poor outcome, 5.41 mmol/L (4.53-6.29) vs. 5.85 mmol/L (5.19–6.50)). ROC curve analysis was also carried out to determine whether *α*-KG levels in C1 could predict poor outcome at 3 months after SAH (Figure 1(h)). We chose glucose levels in B1 as the positive control group. The AUCs for glucose and *α*-KG as predictors of poor outcome were 0.711 and 0.775. There was no significant difference between two biomarkers (*z* = 0.622, *P* = 0.5339).

The article "Alpha-Ketoglutarate Alleviates Neuronal Apoptosis Induced by Central Insulin Resistance through Inhibiting S6K1 Phosphorylation after Subarachnoid Hemorrhage" was published in 2022. Journal: Oxid Med Cell Longev.

### 3.3. Insulin Resistance Occurred in Neurons after SAH

HT22 cells were stimulated with 25 *μ*M Hb. And p-IRS1 (Ser636/639) and IRS1 were detected by WB for 3 h, 6 h, 12 h, 24 h, and 48 h and control groups. It was found that p-IRS1 (Ser636/639) significantly increased at 3 h, 6 h, 12 h, and 24 h after SAH compared with the control group (Figure 2(c)). There was no significant difference in p-IRS1 (Ser636/639) 48 h after SAH compared with the control group (Figure 2(c)). IRS1 showed no significant change at 3 h, 6 h, and 12 h but significantly decreased at 24 h and 48 h (Figure 2(d)). The detection index of IR, p-IRS1 (Ser636/639)/IRS1, was significantly increased 24 h after SAH, which was significantly different from that of control group (Figure 2(e)), indicating that IR appeared at 24 h after SAH. Through qPCR, we examined the expression of IRS1 mRNA in the 12 h, 24 h, and 48 h groups and found that the IRS1 mRNA in the 24 h group was significantly reduced (Figure 2(b)). In addition, the average fluorescent intensity of 2-NBDG was calculated to verify the glucose uptake ability of neuron. Consistent with the Western blot results, the glucose uptake ability of neurons was decreased at 24 h (Figures 2(f) and 2(g)). In conclusion, 24 h was selected as the time point of the follow-up experiment.

### 3.4. *α*-KG Reduced Insulin Resistance of Neurons after SAH and Inhibited the Phosphorylation of S6K1

According to the literature [28], we set three concentration gradients, 0.5 mM, 1 mM, and 2 mM DMKG, respectively. We found that p-IRS1 (Ser636/639) expression level in 1 mM and 2 mM DMKG groups was significantly lower than that in the SAH group. And there was no significant difference compared with the control group (Figure 3(b)). In contrast, p-IRS1 (Ser636/639) levels did not change significantly in the 0.5 mM DMKG group compared with the SAH group (Figure 3(b)). The decrease in IRS1 caused by SAH was recovered only in the 1 mM DMKG group (Figure 3(c)). There was no significant difference in IRS1 expression between the 0.5 mm and 2 mM DMKG groups and the SAH group (Figure 3(c)). Finally, p-IRS1 (Ser636/639)/IRS1 ratios in 0.5 mM, 1 mM, and 2 mM DMKG groups were significantly decreased compared with SAH, and there was no significant difference compared with the control group (Figure 3(d)). In addition, qPCR showed that IRS1 mRNA levels were significantly recovered in the 0.5 mM and 1 mM DMKG groups compared with the SAH group, while there was no significant difference in the 2 mM DMKG group compared with the SAH and Con groups (Figure 3(e)). In addition, the average fluorescent intensity of 2-NBDG was calculated to verify the glucose uptake ability of neuron. Consistent with the Western blot results, the glucose uptake ability of neurons was increased when treated with 0.5 mM, 1 mM, and 2 mM DMKG after Hb stimulation (Figure 3(i)). Therefore, we chose 1 mM DMKG as the drug concentration for subsequent experiments. p-S6K1 (Thr389) level increased markedly after SAH, while that significantly decreased when treat with DMKG (Figure 3(g)). However, S6K1 level did not differ between control, SAH, and SAH+DMKG groups (Figure 3(h)).

The article "Alpha-Ketoglutarate Alleviates Neuronal Apoptosis Induced by Central Insulin Resistance through Inhibiting S6K1 Phosphorylation after Subarachnoid Hemorrhage" was published in 2022. Journal: Oxid Med Cell Longev.

### 3.5. *α*-KG Improved Neuronal Glucose Metabolism and Reduced Neuronal Apoptosis

Glucose transporters in the cell membrane are critical for glucose uptake [34], and glucose transport can serve as an important regulatory point for early apoptotic cascades [6]. We found that the ratio of GLUT4 content in plasma membrane (PM) to total levels of GLUT4 expression in the SAH group was significantly reduced (Figures 4(a) and 4(b)). DMKG could restore the decline of GLUT4 ratio in PM to total levels of GLUT4 after SAH (Figures 4(a) and 4(b)). We further confirmed the glucose uptake capacity of neurons after DMKG administration by calculating the average fluorescent intensity of 2-NBDG (Figures 4(c) and 4(d)). The results showed that the glucose uptake capacity of neurons was consistent with the ratio of GLUT4 expression in PM to total levels of GLUT4. DMKG can reverse the impairment of glucose uptake by neurons after SAH (Figures 4(c) and 4(d)). More importantly, we detected the cell viability of neurons by CCK8 and found that the cell viability decreased significantly after SAH and increased significantly after DMKG administration (Figure 5(a)). Cleaved caspase-3 content (Figures 5(b) and 5(c)) and apoptosis ratio of neurons (Figures 5(d) and 5(e)) increased significantly after SAH. Surprisingly, DMKG could reverse this process. In addition, there were no significant differences in cleaved caspase-3 content and apoptosis ratio between DMKG group and control group. Furthermore, caspase-3 assay kit was used to detect the caspase-3 activity among Con, SAH, and SAH+DMKG groups. The results showed that Hb stimulation could increase caspase-3 activation and did not further increase caspase-3 activation when treated with DMKG (Figure 5(f)).

The article "Alpha-Ketoglutarate Alleviates Neuronal Apoptosis Induced by Central Insulin Resistance through Inhibiting S6K1 Phosphorylation after Subarachnoid Hemorrhage" was published in 2022. Journal: Oxid Med Cell Longev.

### 3.6. *α*-KG Alleviates SAH-Induced Neuronal Apoptosis and Glucose Metabolism Disorder through Inhibiting S6K1 Phosphorylation-Induced IR

We further explored the relationship between IR and apoptosis. The p-IRS1 (Ser636/639)/IRS1 ratios of the SAH group were also significantly increased, while that of the SAH+DMKG group was significantly decreased compared with SAH group (Figure 6(a)). Subsequently, classical inducer of insulin resistance PA was used to upregulate S6K1 and induce IR. There is significantly upregulation of p-S6K1 (Thr389) and p-IRS1 (Ser636/639)/IRS1 in the PA group (Figure 6(a)). More importantly, the content of p-S6K1 (Thr389) and the ratio of p-IRS1 (Ser636/639)/IRS1 in the SAH+DMKG+PA group increased again, which was significantly higher than that in the SAH+DMKG group (Figure 6(a)). Compared with the control group, PA significantly reduced the ratio of GLUT4 expression in PM to total levels of GLUT4 expression (Figure 6(b)) and inhibited the glucose uptake of neurons (Figure 6(c)). Cleaved caspase-3 of neurons in the PA group was significantly higher than that in the control group (Figure 6(d)). Flow cytometry showed that the proportion of early apoptosis was significantly increased in the PA group (Figure 6(e)). Similarly, Hb stimulation also significantly increased cleaved caspase-3 and the proportion of neuronal apoptosis (Figures 6(d) and 6(e)). Moreover, the mitigative effect of DMKG on the apoptosis induced by Hb stimulation was inhibited by PA (Figures 6(d) and 6(e)). In short, in the SAH+DMKG+PA group, the ratio of GLUT4 expression in PM to total levels of GLUT4 expression and the average fluorescent intensity of 2-NBDG within neurons were significantly decreased (Figures 6(b) and 6(c)), and cleaved caspase-3 and apoptosis rates were significantly increased (Figures 6(d) and 6(e)).

### 3.7. *α*-KG Inhibited S6K1 Activity

Recent studies have found that S6K1 is overactivated in SAH and reaches its peak at 24 h [35]. S6K1 plays an important role in driving IR [20]. Moreover, deletion of S6K1 can reduce p-IRS1 (Ser636/639) and increase insulin sensitivity in obese mice [21]. Therefore, we hypothesized that the overactivated S6K1 after SAH promotes insulin resistance in brain tissues. We hypothesized that *α*-KG might inhibit IR by inhibiting S6K1 activation. We performed molecular docking to predict the binding mode of *α*-KG to S6K1. The crystal structure of human S6K1 protein was downloaded from PDB (PDB ID: 4RLP). The 3D structure of small molecule alpha-ketoglutarate (Figure 7(a)) was downloaded from PubChem database. The energy was minimized under MMFF94 field. In this study, the AutoDock Vina 1.1.2 software was used for molecular docking. Before docking, PyMOL 2.5 was used to process all receptor proteins, including removing water molecules, salt ions, and small molecules. Then, the docking box was set. The PyMOL software was used to define the centroid of the crystal ligand as the center of the docking box. The side length of the cubic box was set as 25 angstroms. In addition, all processed small molecules and receptor proteins were converted to the required PDBQT format by AutoDock Vina 1.1.2 using ADFRsuite 1.0. During interconnection, the global search detail is set to 32, and other parameters retain default settings. The docking conformation with the highest output score was thought to be the binding conformation. And the docking results of PyMOL 2.5 were finally used for visual analysis. We found that the small molecule alpha-ketoglutarate binds to the ATP pocket of the protein, and the carboxyl group on the molecule forms hydrogen bonding with LEU-175 on the hinge of the S6K1 protein. In addition, it can also be seen from the figure that small molecules can form hydrophobic interactions with LEU-175 and THR-235 on the protein. The result of molecular docking and the ability of *α*-KG to decrease the phosphorylation of S6K1 suggest that S6K1 is the molecular target of *α*-KG (Figures 3(f), 6(a), and 7(a)). Therefore, we conducted an in vitro kinase assay to further verify the interaction of *α*-KG and S6K1. We found that *α*-KG indeed inhibited the activity of recombinant S6K1 (Figure 7(b)). As a comparison, the S6K1-specific inhibitor, PF-4708671 (MedChemExpress, HY-15773), at the concentration of 10 *μ*M inhibited S6K1 activity by 65.3%.

The article "Alpha-Ketoglutarate Alleviates Neuronal Apoptosis Induced by Central Insulin Resistance through Inhibiting S6K1 Phosphorylation after Subarachnoid Hemorrhage" was published in 2022. Journal: Oxid Med Cell Longev.

### 3.8. *α*-KG Alleviated Neuronal Apoptosis after SAH in Mice

We further detected whether *α*-KG could also alleviate neuronal apoptosis in SAH mice. The SAH group had significantly higher NeuN^+^ TUNEL^+^ proportion than those in the sham group (*n* = 3, 5.71 ± 2.51% in the sham group vs. 57.79 ± 4.48% in the SAH group). Mice treated with *α*-KG had remarkably lower NeuN^+^ TUNEL^+^ proportion than those in the SAH group (*n* = 3, 57.79 ± 4.48% in the SAH group vs. 22.05 ± 4.68% in the SAH + DMKG group) (Figures 8(a) and 8(b)). There was no difference between sham group and SAH+DMKG group. Besides, the expression of cleaved caspase-3 was decreased when treated with *α*-KG (Figure 8(c)).

## 4. Discussion

The elevation of blood glucose caused by SAH seriously affects the prognosis of patients. Studies have shown that IR is the direct cause of such glucose metabolism disorder [7–10]. Insulin binding to insulin receptors promotes IRS phosphorylation at different tyrosine sites, thereby activating the PI3K-Akt pathway. Abnormal phosphorylation of serine residues inhibits the PI3K-Akt pathway [22]. As a key product of TCA, *α*-KG has been reported to improve insulin sensitivity and reduce blood glucose in obese mice [27, 28]. Our study focused on the mechanism of *α*-KG inhibiting IR after SAH and identified S6K1 as its molecular target. Our study provides new insights into the occurrence and compensation of IR after SAH.

Insulin selectively acts through IRS1 in the cerebellar cortex and hippocampus of adults [18]. Talbot et al. pointed out that p-IRS1 (Ser636/639) expression was generally elevated in hippocampal neurons of AD patients, and p-IRS1 (Ser636/639) could serve as a potential biomarker of IR in brain tissues [18]. The ratio of IRS serine phosphorylation to IRS tyrosine phosphorylation is proposed as a marker of peripheral and cerebral IR. Kellar and Craft and Peng et al. took p-IRS1 (Ser636/639)/IRS1 as a marker of IR [22, 23]. Based on the above research background, p-IRS1 (Ser636/639)/IRS1 was finally selected as the marker of IR. Previous studies on IR after SAH have focused on the changes of systemic insulin sensitivity in SAH patients [7–10], but there is still a lack of studies on IR in local brain tissues after SAH. Scherer et al. thought that cerebral IR occurred before systemic IR [36], which attracted our attention to the importance of IR in brain tissue after SAH. Neurons consume 80-85% of the energy used by brain tissue. Moreover, ATP required by neurons is almost produced by glucose metabolism [14, 37]. Therefore, in this study, an in vitro model of SAH was established by stimulating neurons with Hb. And a preliminary study found that IR occurred in neurons after 24 h Hb stimulation.

For hyperglycemia after SAH, the effects of insulin treatment are not satisfied even with a high risk of hypoglycemia [8]. Targeted treatment of central IR seems to be a better way to improve energy metabolism disorders with a lower risk of hypoglycemia [36]. Therefore, IR of brain tissue after SAH may be a reliable way to improve systemic glucose metabolism. The transient increase in blood glucose after SAH [7–10] suggests that there may be a mechanism to alleviate this glucose metabolism disorder in human body. We found that the CSF *α*-KG levels increased over time after SAH. As a key biological compound, *α*-KG plays an important role in different metabolic and cellular pathways [38, 39]. Glutamic acid dehydrogenase can convert glutamic acid to *α*-KG. And increased *α*-KG can promote insulin secretion [40]. At the same time, *α*-KG is involved in the catabolism of branched chain amino acids (BCAA), and the inhibition of BCAA catabolism is related to the occurrence of IR [41]. In addition, *α*-KG has been shown to improve insulin sensitivity and reduce blood glucose in obese mice [27, 28]. Our results showed that neuronal IR induced by Hb stimulation could inhibit the expression of GLUT4 in the cell membrane and reduce neuronal glucose uptake. However, *α*-KG could significantly alleviate this decrease, increase GLUT4 level in neuron membrane, and promote the glucose uptake of neurons.

The article "Alpha-Ketoglutarate Alleviates Neuronal Apoptosis Induced by Central Insulin Resistance through Inhibiting S6K1 Phosphorylation after Subarachnoid Hemorrhage" was published in 2022. Journal: Oxid Med Cell Longev.

S6K1 is a recognized signal molecule in the insulin signaling pathway PI3K/AKT/mTOR which plays an important role in the pathogenesis of type 2 diabetes [42]. Hypertrophic phosphorylation of p-S6K1 (Thr389) reduces insulin sensitivity by promoting p-IRS1 (Ser636/639) expression. Conversely, S6K1 knockout reduced p-IRS1 (Ser636/639) expression and restored insulin sensitivity in obese mice. Therefore, S6K1 may play a nonnegligible role in the development of IR and is an important drug target for IR treatment [21]. Talbot et al. pointed out that the elevation of p-IRS1 (Ser636/639) in hippocampal neurons of AD patients was positively correlated with the activation of mTOR [18]. S6K1, as a serine/threonine protein kinase downstream of mTOR, is likely to be involved in the upregulation of p-IRS1 (Ser636/639) in hippocampal neurons. You et al. found that S6K1 was overactivated in the in vitro model of SAH and reached a peak at 24 h [35], which was consistent with the results of the in vitro model of SAH established by Hb stimulation of neurons in this study. Our study found that *α*-KG had an interaction with S6K1; that is, *α*-KG could inhibit both the phosphorylation of S6K1 and the IR after SAH. In addition, the inhibitory effect of *α*-KG on IR was negatively regulated by PA through activation of S6K1, suggesting that *α*-KG could be used as a potential inhibitor of S6K1 to suppress IR after SAH by targeting the phosphorylation of S6K1. What is more, we found that *α*-KG could dock ATP-binding pockets in the S6K1 enzyme activity center, suggesting a potential binding mode between *α*-KG and S6K1, and we proved that *α*-KG can inhibit S6K1 activity in vitro kinase assay.

The article "Alpha-Ketoglutarate Alleviates Neuronal Apoptosis Induced by Central Insulin Resistance through Inhibiting S6K1 Phosphorylation after Subarachnoid Hemorrhage" was published in 2022. Journal: Oxid Med Cell Longev.

Glucose transport and metabolism may be crucial regulatory points in the early apoptotic cascade. Decreased cellular ATP levels induced by impaired glucose transport are thought to participate in neuronal apoptosis [6]. Liu et al. found that small compound inhibitors of basal glucose transport inhibit cell proliferation and induce apoptosis in cancer cells via glucose-deprivation-like mechanisms [43]. Rizzo et al. studied the mechanisms of neuronal death in ischemic stroke by establishing an in vitro model of oxygen and glucose deprivation and found that continuous oxygen and glucose deprivation significantly reduced neuronal activity and increased neuronal death [44]. It has been reported that type 2 diabetes rats have impaired learning and memory function due to apoptosis of hippocampal neurons. However, this cognitive impairment is alleviated by inhibiting IR [45, 46]. Similarly, we also found that *α*-KG reduced the apoptosis of neurons after SAH both in vitro and in vivo and promoted glucose uptake of neurons in vitro study. More importantly, the role of *α*-KG in alleviating neuronal apoptosis was inhibited by PA's reduction of glucose uptake through activation of S6K1. Likewise, some researchers have found that inhibition of S6K1 activation induced by SAH can increase the number of viable neurons [35]. These results suggest that *α*-KG can inhibit the IR induced by S6K1 activation, promote the levels of GLUT4 in cell membrane, and increase cellular glucose uptake, thereby alleviating the early apoptosis of neurons (Figure 9).

According to literature reports, increased phosphorylation of AMPK could promote the increase of *α*-KG [47]. Phosphorylation of AMPK increased after SAH [48], which could well explain the increased *α*-KG level of cerebrospinal fluid in SAH patients in this study. In addition, this study also found that protein and mRNA levels of IRS1 in neurons decreased significantly after SAH. Similar results were consistent with those in AD [15]. Exogenous *α*-KG administration could restore this reduction. Based on the fact that *α*-KG acts as a common substrate for more than 60 dioxygenases including TET family [49], recent studies have demonstrated that *α*-KG can increase the demethylation of Prdm16 promoter through TET family, upregulate Prdm16 gene, and ultimately increase insulin sensitivity and regulate blood glucose [28]. We speculate that *α*-KG in SAH may be involved in the demethylation of IRS1 promoters through the TET family, which we plan to further verify in subsequent studies.

The article "Alpha-Ketoglutarate Alleviates Neuronal Apoptosis Induced by Central Insulin Resistance through Inhibiting S6K1 Phosphorylation after Subarachnoid Hemorrhage" was published in 2022. Journal: Oxid Med Cell Longev.

## 5. Conclusion

In conclusion, our studies found a remarkable increase of *α*-KG in CSF of SAH patients, which could alleviate IR induced by SAH, and confirmed *α*-KG as a potential inhibitor of S6K1 in vitro. *α*-KG inhibits the increase of p-IRS1 (Ser636/639)/IRS1 caused by the increase of S6K1 phosphorylation induced by Hb stimulation, thereby increasing the expression of GLUT4 in the cell membrane, increasing glucose uptake, and ultimately alleviating neuronal apoptosis.

## Figures and Tables

**Figure 1:** *α*-KG not only remarkably increased after SAH but also predicted the prognosis of SAH patients. (a) *α*-KG levels in cerebrospinal fluid in the control group and 1-3 days after subarachnoid hemorrhage (C1) and 5-7 days after subarachnoid hemorrhage (C2) (Kruskal-Wallis); 21 patients who have both C1 and C2 were compared by paired tests (paired *t*-test). (b) Glucose levels of 1-3 days after hemorrhage (B1), 5-7 days after hemorrhage (B2), and the day before discharge (Kruskal-Wallis); 21 patients who have both B1 and B2 were compared by paired tests (paired t-test). (c, d) The levels of *α*-KG in cerebrospinal fluid 1-3 days and 5-7 days after hemorrhage in the two groups with different outcomes (unpaired *t*-test, *F* = 1.51; *F* = 2.28). (e, f) Blood glucose levels 1-3 days and 5-7 days after bleeding in patients with different outcomes (unpaired *t*-test, *F* = 1.78; *F* = 1.81). (g) The correlation analysis and stratified analysis between *α*-KG levels in C1 and HUNT-HESS score (Spearman analysis). (h) Receiver operating characteristic curves for *α*-KG levels in C1 and glucose levels in B1 (^∗^*P* < 0.05; ^∗∗^*P* < 0.01; ns: no significance).

**Figure 2:** IR occurred in neurons after SAH. (a, c) Expression of p-IRS1 (Ser636/639) with or without Hb stimulation for 3 h, 6 h, 12 h, 24 h, and 48 h (one-way ANOVA, *F* = 19.42). (b) mRNA expression of IRS1 with or without Hb stimulation for 12 h, 24 h, and 48 h (one-way ANOVA, *F* = 16). (a, d) Expression of IRS1 with or without Hb stimulation for 3 h, 6 h, 12 h, 24 h, and 48 h (one-way ANOVA, *F* = 4.79). (a, e) p-IRS1 (Ser636/639)/IRS1 ratio after Con and Hb stimulation for 3 h, 6 h, 12 h, 24 h, and 48 h (one-way ANOVA, *F* = 4.43). (f, g) Glucose uptake ability was calculated by the average fluorescent intensity of 2-NBDG, bar = 200 *μ*m (one-way ANOVA, *F* = 14.15) (^∗^*P* < 0.05, ^∗∗^*P* < 0.01).

**Figure 3:** *α*-KG inhibited IR after SAH. (a, b) p-IRS1 (Ser636/639) levels in the control, SAH, and DMKG groups (one-way ANOVA, *F* = 12.51). (a, c) IRS1 levels in the control, SAH, and DMKG groups (one-way ANOVA, *F* = 4.67). (a, d) p-IRS1 (Ser636/639)/IRS1 ratio of the control, SAH, and DMKG groups (one-way ANOVA, *F* = 32.42). (e) IRS1 mRNA levels in the control, SAH, and DMKG groups (one-way ANOVA, *F* = 6.168). (f, g) p-S6K1 (Thr389) level of the control, SAH, and SAH+DMKG groups (one-way ANOVA, *F* = 17.56). (f, h) S6K1 level of the control, SAH, and SAH+DMKG groups (one-way ANOVA, *F* = 1.05). (i) Glucose uptake ability was calculated by the average fluorescent intensity of 2-NBDG, bar = 200 *μ*m (one-way ANOVA, *F* = 44.86) (^∗^*P* < 0.05, ^∗∗^*P* < 0.01).

The article "Alpha-Ketoglutarate Alleviates Neuronal Apoptosis Induced by Central Insulin Resistance through Inhibiting S6K1 Phosphorylation after Subarachnoid Hemorrhage" was published in 2022. Journal: Oxid Med Cell Longev.

**Figure 4:** *α*-KG improved glucose metabolism of neurons after Hb stimulation. (a, b) The ratio of GLUT4 expression in plasma membrane to total levels of GLUT4 expression in the control, SAH, and SAH+DMKG groups (one-way ANOVA, *F* = 7.89). (c, d) Glucose uptake ability was calculated by the average fluorescent intensity of 2-NBDG, bar = 50 *μ*m (one-way ANOVA, *F* = 11.78) (^∗^*P* < 0.05, ^∗∗^*P* < 0.01).

**Figure 5:** *α*-KG alleviated neuronal apoptosis induced by SAH. (a) CCK-8 detection of neurons in the control, SAH, and SAH+DMKG groups (one-way ANOVA, *F* = 17.74). (b, c) Expression of neuron cleaved caspase-3 in the control, SAH, and SAH+DMKG groups (one-way ANOVA, *F* = 28.54). (d, e) Neuronal apoptosis was detected by flow cytometry in the control, SAH, and SAH+DMKG groups (one-way ANOVA, *F* = 11.75). (f) Caspase-3 assay kit was used to detect the caspase-3 activity (one-way ANOVA, *F* = 45.36) (^∗^*P* < 0.05, ^∗∗^*P* < 0.01).

**Figure 6:** *α*-KG could reduce neuronal apoptosis by inhibiting IR. (a) Level of p-IRS1 (Ser636/639), IRS1, p-IRS1 (Ser636/639)/IRS1 ratio, and p-S6K1 (Thr389) in control, Con+PA, SAH, SAH+DMKG, and SAH+DMKG+PA groups (one-way ANOVA, *F* = 10.82; *F* = 10.76; *F* = 17.02; *F* = 15.73). (b) The ratio of GLUT4 expression in plasma membrane to total levels of GLUT4 expression in control, Con+PA, SAH, SAH+DMKG, and SAH+DMKG+PA groups (one-way ANOVA, *F* = 72.93). (c) Glucose uptake ability was calculated by the average fluorescent intensity of 2-NBDG in the control, Con+PA, SAH, SAH+DMKG, and SAH+DMKG+PA groups, bar = 200 *μ*m (Kruskal-Wallis). (d) Expression of cleaved caspase-3 in the control, Con+PA, SAH, SAH+DMKG, and SAH+DMKG+PA groups (one-way ANOVA, *F* = 9.52). (e) Proportion of early apoptotic detected by Annexin V-FITC/PI staining (one-way ANOVA, *F* = 39.1) (^∗^*P* < 0.05, ^∗∗^*P* < 0.01).

**Figure 7:** (a) The binding mode of alpha-ketoglutarate to S6K1 protein was obtained based on docking. The left picture is the overall view, and the right picture is the local view. Blue stick is the small ligand molecule, light blue cartoon is the protein, gray dotted line represents hydrophobicity, and yellow dotted line represents hydrogen bonding. (b) The ability of *α*-KG to inhibit S6K1 activity was assayed by ADP-Glo™ kinase kit (one-way ANOVA, *F* = 553.81) (^∗∗^*P* < 0.01).

The article "Alpha-Ketoglutarate Alleviates Neuronal Apoptosis Induced by Central Insulin Resistance through Inhibiting S6K1 Phosphorylation after Subarachnoid Hemorrhage" was published in 2022. Journal: Oxid Med Cell Longev.

**Figure 8:** *α*-KG alleviated neuronal apoptosis after SAH in mice. (a, b) The TUNEL images and the whole-brain NeuN^+^ TUNEL^+^/NeuN^+^ proportion, bar = 1 mm (one-way ANOVA, *F* = 44.15). (c) Expression of cleaved caspase-3 in the sham, SAH, and SAH+DMKG groups (one-way ANOVA, *F* = 9.44).

**Figure 9:** After SAH, mTOR/S6K1 pathway is activated in neurons, which inhibits the normal phosphorylation of IRS1, ultimately inhibits translocation of GLUT4, and reduces the expression of GLUT4 in neuron membrane. DMKG can relieve the inhibition of IRS1 and its downstream pathways after SAH by inhibiting the mTOR/S6K1 pathway.

**Table 1:** Primer sequences and antibodies involved.

qPCR	IRS1-F	CGATGGCTTCTCAGACGTG
qPCR	IRS1-R	CAGCCCGCTTGTTGATGTTG
Antibody	p-IRS1 (Ser636/639)	Cell Signaling Technology (#2388)
Antibody	IRS1	Cell Signaling Technology (#2382)
Antibody	GLUT 4	Proteintech (66846-1-lg)
Antibody	Cleaved caspase-3	Abcam (ab2302)
Antibody	p-S6K1 (Thr389)	Proteintech (28735-1-AP)
Antibody	S6K1	Proteintech (14485-1-AP)
Antibody	Actin	Abmart (M20011)
Antibody	Tubulin	Abmart (M30109)

**Table 2:** Univariate analysis comparing patients with poor and good 3-month outcomes.

Variable	MRS, 0-2	MRS, 3-6	*P* value
Males/females	16 (32%)/23 (46%)	3 (6%)/8 (16%)	0.498
Mean age in years	57 (47-67)	63(53-73)	0.083
Hypertension	20 (40%)	8 (16%)	0.306
DSA			0.174
Positive	31 (62%)	11 (22%)	
Negative	8 (16%)	—	
Aneurysm location			0.647
Anterior	25 (50%)	9 (18%)	
Posterior	4 (8%)	2 (4%)	
Multiple aneurysms	2 (4%)	—	
Admission Hunt-Hess score			0.306
1	9 (18%)	2 (4%)	
2	20 (40%)	3 (6%)	
3	9 (18%)	5 (10%)	
4	1 (2%)	1 (2%)	
5	—	—	

MRS: Modified Rankin Scale; DSA: digital subtraction angiography.

## Data Availability

The authors confirm that the data involved are available upon reasonable request.
